This article has been retracted.

# Promotion and Protection of Feminism Creativity for Public Environment: The Integration of Ecofeminism and Public Environment

**DOI:** 10.1155/2022/5706699

**Published:** 2022-11-21

**Authors:** Wanjin Dong, Soonbae Kim

**Affiliations:** ^1^Nanyang Medical College, Nanyang 473000, China; ^2^Chungbuk National University, Chungbuk 28644, Republic of Korea

## Abstract

Each of us leaves a trace of our consumption on the environment. Take a step back, though, and consider how much influence people have had on the Earth. The Anthropocene, sometimes known as the era of humans, refers to how significantly we have changed the Earth's systems. This is the grand view of humanity's impact on the Earth. In this article, we plan to introduce and explain ecofeminism. Because of the natural connection with nature and the social role as housekeepers, women often have empathetic power when expressing their demands for the public environment, thus becoming a vital force in public environmental protection. Facing the public environmental forces spurting from ecofeminism, we study the dissemination of ecofeminism with the help of mass media. However, in present-day China, as pointed out by ecofeminism, the predatory exploitation of nature and the catastrophic killing of plants and animals make the fate of women challenging to control. Therefore, we study the theory of multicultural ecofeminism and public environmental protection. Finally, based on the integration of ecofeminism and the public environment, we interpret Lawrence's famous work, Sons and Lovers, and analyze the relationship between men and women and the public environment in this work from the perspective of ecofeminism. In human socialization, ecofeminism has provided strong support for protecting the public environment, and at the same time, it has also improved.

## 1. Introduction

In the 1970s, ecofeminism emerged with the environmental movement in Western society and developed rapidly in the West. Ecofeminism maintains that the question of “nature” and “woman” is naturally related. Its core argument is that there is a historical isomorphism between “belittling nature” and “belittling women” [1, 2]. The reason why ecofeminists pay attention to “nature” is that they try to construct a new relationship between man and nature by analyzing the root of the contradiction between man and nature, so as to realize the liberation of nature and women [3]. Certainly, ecofeminists try to overcome the ecological crisis faced by mankind with the restoration of “female principles.” The emergence of ecofeminism has led to a green revolution [4–6]. It reveals the connections between the myriad forms of oppression rooted in man's efforts to control nature, especially the oppression of women. To eliminate the inequality imposed on women by the patriarchal society, it struggles to give women the same free and equal social power as men. It strives to realize the cooperation and joint development between men and women. The essence of ecofeminism points to the protection of harmonious cultural ecology and cultural environment. Its activists strive for equality between men and women in the sense of cultural ecology and environmental protection. They not only achieve equality in social status and human rights but also realize women's reasonable status and legal rights in personality and culture.

Like other feminists, ecofeminism strives for the equality and harmonious development of men and women in society. In 1974, Françoise d'Eaubonne first used ecofeminism and revealed that the oppression of women by patriarchy was directly related to the oppression of nature, including historical, empirical, symbolic, and theoretical connections, which led to an ecological and environmental humanistic revolution [7–10]. In ecofeminism, as shown in Figure 1, the prefix eco comes from ecology or the study of living organisms and their environment, and feminism in its basic sense relates to the advocacy for gender equality in women's rights. Ecofeminists have sharply criticized and sought to subvert the patriarchy that caused these oppressions and the erroneous concept of duality between nature and culture, pointing out that it is a feature of patriarchal society. They extend the inequality of hierarchy between men and women to the separation of culture and nature and the difference of opposing hierarchies. Patriarchy, just like the oppression and coercion of women, starts to plunder and control nature to show the superiority and hegemony of patriarchy.

Ecofeminism is richer than any other branch of feminism in that it strives to expose the connections between the myriad forms of oppression rooted in man's efforts to control nature. Ecofeminism is also a decisive understanding of feminism and environmental ethics [11–15]. It discovers the tragic reality of the patriarchal misconception that separates animals from humans, men, and women. There are many branches of ecofeminism, which can be divided into two types: the ecofeminism of social constructionism and the ecofeminism of naturalism. The so-called ecofeminists of social constructivism regard the connection between women and nature, men and social culture as their subordination to women (or women to men) and human predation of nature. They believe this idea of patriarchy is so powerful that women, like men, believe that women belong only to the private sector, where they use their hands and thoughts to raise their children. While men belong to the public domain, where productive and creative work takes place; men use their machines and computers to build society. For feminists of social constructivism, the position taken by some challenges the idea that women are detached from the limited connection between nature and reproduction, that there is absolutely no idea that nature is inferior to culture, or that reproduction is less valuable than production. The special qualities of women stem from their biological connection to the reproduction process of nature, not from the denial of their connection to nature. Women should unwaveringly adhere to nature rather than culture. Reproduction, not production, is an absolute necessity for life [16–19]. Ecofeminism believes that women tend to value relationships and special individuals because of their nature and female experience. They emphasize care, nurturing, and affection, and they strive to reset conflicting and individual claims in a cooperative and communal way.

The theoretical and practical significance of ecofeminism lies in the following: First, it tries to end the sexist oppression and discrimination against women and nature. Androcentrism includes any concept that controls the dominance or subordination of women, which results in the existence of oppression of sexist. Additionally, sexist bias exists in language as well as in many other fields, including employment, education, and so on, and the erroneous thoughts and realities that separate and oppose men from women, nature, and culture must be completely eliminated. Second, ecofeminism tries to safeguard the potential of women. It further points out the patriarchy's discrimination against nature, biology, and women, which separates and antagonizes them from the human social culture-men. Third, ecofeminism strives to eliminate such inequality and unreasonable reality, strives for social and cultural power, and creates equal and harmonious relations and culture. In essence, it is a cultural, ecological public environment protection theory. The contributions of this study are summarized as follows:

1. Facing the public environmental forces spurting from ecofeminism, we study the dissemination of ecofeminism with the help of mass media
2. We study the theory of multicultural ecofeminism public environmental protection
3. Based on the integration of ecofeminism and public environment, we interpret Lawrence's famous work, Sons and Lovers, and analyze the relationship between men, women, and public environment in this work from the perspective of ecofeminism

The rest of the article is organized as follows. In Section 2, the ecofeminist movement and dissemination of ideological trend helped by mass media is studied.  Section 3 studies multicultural ecofeminist public environmental protection. In Section 4, the ecofeminism in Sons and Lovers is interpreted.  Section 5 concludes this article.

## 2. Ecofeminist Movement and Dissemination of Ideological Trend Helped by Mass Media

Before the formation of social movements, women had already been deeply involved in the field of public environment due to ontological experiences and concern for family life [20–25]. In the 1960s, in the United States, women started their own environmental activism to address the health and public environment problems they and their families faced. At the beginning, faced with the cruel behavior of human beings, especially men, who randomly hurt animals in the name of developing science and technology, women instinctively linked the fate of animals with their own fate and called for the protection of animals' survival rights. Afterwards, women's concerns about the public environment directly prompted their participation in urban environmental reform activities. During this period, most of the women tended to achieve environmental protection through political channels. They were committed to promoting environmental laws and administrative orders to ensure healthy public environment for their families. Out of maternal concern for the public environment and concern for family life, women instinctively raised their voices for improving the public environment by conducting investigations, making speeches and seeking the help of government departments by making use of their influence, mobilizing the participation of public people in improving public environment from an individual perspective, and eventually pushing for government environmental policy and laws. These kinds of women's conscious behaviors directly popularized and spread the concept and knowledge of protecting urban health. Using gender as a vantage point, ecofeminism examines the conditions that cause and perpetuate the subordination of both women and nature. It can be thought of as a lens for examining intersections of oppression; harmful practices that exploit the environment and social structures that oppress women among other groups have an overlap, and that is what ecofeminism is all about, as shown in Figure 2.

Women's protection of the public environment shows their close connection with nature and strengthens their social role as “family caregivers,” but at the same time, they are satirized and attacked by the patriarchal civilization. They believe that these women's environmental behavior is purely out of personal emotions and concern for their individual lives, lacking rationality and technology, and lacking sublime and applicability [26–28]. In the face of all kinds of criticism and scrutiny, female public environmental protection activists with ecofeminist consciousness began to realize that women's marginal status is the main reason behind men despising and belittling women's environmental protection behavior. In a male-centered patriarchal society, women's true meaning and value are diminished or even totally denied. They are imprisoned in the private sphere of family life for a long time, unable to participate in the discussion and decision-making of public affairs, and eventually become victims of male activities just like nature. Therefore, ecofeminism gradually shows a strong color of publicity, which emphasizes that women must act against the oppression of patriarchal social culture, change their position, seek equal social status and speech rights with men, and then gain a place in the public sphere. As there is a natural affinity between women and nature, public environmental problems can link family life and public society. Hence, ecofeminists consciously take the intervention of environmental issues as an important way for women to resist male chauvinism and compete for public power.

At the same time, as the disadvantages of industrial civilization become more and more obvious and the development of mass media becomes more and more mature, environmental problems begin to gain more attention in the mass media. Media disseminates and reports environmental events and information in a popular way, widely popularizing the concept of environmental protection. They purposefully stimulate and guide public sentiment and public opinion, thus influencing the progress of environmental events and environmental movement. Under the influence of mass media, social resources have been highly mobilized and integrated, and civil environmental protection forces have effectively united and entered the environmental movement, thus forming a wave of social movement, which has a crucial impact on the formulation of government public environmental policies and the implementation of environmental protection measures.

Aware of the media's communication advantages, ecofeminists began to actively use the mass media to expand their influence. They consciously seized the media's right of speech, sought resource mobilization and support nationwide, and infected other classes and groups of society with a positive attitude to protect the environment, resulting in universal linkage and imitation of social effects. In this process, driven by some women scholars and sportsmen, the expression of ecofeminism has become more and more mature, and the perspective of ecofeminism has begun to become familiar to ordinary people through the mass media, and is gradually becoming known to the public through the mass media.

For ecofeminists, the public environment communication activities carried out by means of mass communication finally expanded the activities with self-liberation significance to a broader public stage. With the reports and propaganda of mass media, women show advanced environmental concepts, keen perception, and strong environmental protection power in the field of social life, which also makes the movement of women outside the private field prominent enough to be recognized by the public [29, 30]. At the same time, the success of these campaigns has also accumulated experience for women public environmentalists in developing feminist ecology. This is because women's involvement in public environmental issues, on the one hand, enhances and amplifies their advantages and abilities in perceiving environmental hazards and achieves the initial goal of public environmental protection. On the other hand, it is also an essential way for women to participate in the public sphere and compete with the male-centered social structure and institutional culture.

In all kinds of public environment communication activities developed through the mass media, women have actually experienced a tremendous change in environmental perspective and motivation. From the very beginning, they only concerned themselves and their families' living environment, and then actively helped other people in society to solve the public environmental problems. In this process, women are no longer trapped in their private lives, but become important participants in the public sphere and have a significant impact on social development. The success of this activity also confirms the core concept of feminist ecology, that is, women construct a way to resist the gender oppression of patriarchal society in their campaign to protect the public environment.

Driven and motivated by mass media and women, more and more ordinary people begin to pay attention to public health and public environment and try to participate in the process of public environment. With the continuous exposure and development of mass media, the resources and forces of environmental protection in society have been highly mobilized and integrated to the maximum extent, thus forming a wave of social movement. Ecofeminism and public environmental communication gradually break through the limitations of groups and go to the public arena, becoming a common topic in the public field. At this time, the social movement initiated by the women's public environmental protection movement and other groups resisting the oppression of social system began to have a theoretical and practical connection, and the feminist ecological trend of thought was ready to give theoretical support to the public environmental justice movement.

Originally, the patriarchal society oppressed not only women and nature, but also vulnerable groups such as colored people and low-income people. Like women, they are also excluded from the public sphere, lack the corresponding science and technology and the opportunity to participate in public decision-making, and thus cannot enjoy equal environmental welfare and become victims of the public environmental crisis. In addition, when faced with environmental problems, the cries for help from other vulnerable groups like women are often not taken seriously. Ordinary people's accusations about chemical pollution or other public environmental problems are considered to be too emotional or ignorant. Their beliefs and voices expressed in public forums are often defined by government officials as unseemly or inappropriate.

## 3. Multicultural Ecofeminism Public Environmental Protection

In the process of China's rapid modernization, the status of women has witnessed a downward trend. Although they have participated in a lot of work, the status and role of women have not been recognized much, and women's employment and development are also faced with difficulties [31]. In present-day China, as ecofeminism points out, the fate of women has become challenging to master due to the predatory development of nature and the catastrophic slaughter of animals and plants. Therefore, we urgently need the rapid rise and development of ecofeminism and, more importantly, emphasize the essence and direction of ecological feminism, cultural ecology, and cultural environmental protection. Cultural ecology and environmental protection should not only overturn and adjust the binary opposition between men and women, but also between culture and nature and between spirit and body, and achieve integration and perfection through humanistic revolution.

In thousands of years of human history, patriarchy has dominated the power of human culture, vigorously excluded the status of women in culture, completely denied the role of women in cultural creation, and greatly persecuted the cultural ecological balance of human society. Ecofeminism reveals the correlation between nature's oppression and women's oppression, and indicates men's coerciveness and hegemonic status in social culture. This kind of cultural monopoly is the characteristic of patriarchy, which produces a series of patriarchal value systems and patriarchal social structures. Men are dominant and superior, while women are subordinate and inferior. The “three obedience and four virtues” of the Chinese feudal society denied the status and identity of women as social and cultural subjects, and only regarded women as a tool for bearing children and carrying on the family line, depending on men.

Ecofeminism is a multicultural ecological public environment protection theory, which points out the crisis and trap that human beings are facing in public environment [32]. Ecofeminism has made positive efforts in multiculturalism. It not only pays attention to women's human and cultural ecological public environment, but also emphasizes the cultural ecological environmental protection of women's spirit. There are three aspects of women's spiritual and cultural ecological protection. (1) the spirit of promotion, (2) paying attention to the cultivation of inner nature, and (3) having a conscious sense of regeneration. In essence, the combination of spiritual and social dimensions is a conscious act to protect the cultural ecological environment.

Harmonious cultural ecological environmental protection is a harmonious cooperative system of equal symbiosis formed by the internal and external elements and their interaction of the humanistic interactive system consciously realized through humanism. Cultural ecology is a world created for humans, more systematic than nature or conceptual natural ecology. It not only includes the transformation of people's ideological and moral quality, but also includes people's scientific and cultural quality. It has the tradition of thousands of years of historical and cultural accumulation, but also faces the impact of foreign culture, with the important task of cultural innovation.

## 4. Ecofeminist Interpretation of Sons and Lovers

### 4.1. Sons and Lovers Review

Author, poet, and essayist David Herbert Lawrence was born in England. His works are primarily based on his early experiences in Nottinghamshire, which had a significant impact on his life. His work reflects modernity's and industrialization's dehumanizing effects. Lawrence had spent his entire life being concerned about human sexuality; emotional health; and relationships between men, women, and nature (public environment). His novels and short stories have been reprinted in huge numbers and translated into a variety of languages around the world. Sons and Lovers is still one of the most popular works among the readers [33].

Sons and Lovers, first published in 1913, is today regarded as Lawrence's early masterpiece and semiautobiographical novel. Furthermore, it is usually regarded as the first significant novel to depict the lives of English working-class people. It came ninth on a list of the 100 best novels in English of the 20th century by the Modern Library in 1999. According to Lawrence, the novel's goal is to depict the tragedy of all British kids of his generation. Chinese critics and scholars have used a variety of theoretical frameworks to understand *Sons and Lovers*, including postmodernism, Freudian psychoanalysis, archetypal criticism, ethical critique, and feminist criticism.

Sons and Lovers is examined from an ecofeminist viewpoint in this section. Public environment and women are intrinsically intertwined, according to ecofeminism, and patriarchy is their common source of domination. The most important contribution of ecofeminism is the recognition of various socioeconomic injustices and oppressions caused by patriarchal ideals.

With its descriptions of public environment, various female characters, and the disharmonious relationship between men and women, Lawrence convincingly conveys the permanent traumas of public environment, the suppressed helpless existence of women, and the associated sorrow of men in Sons and Lovers. Lawrence's statements are all reflective of his ecofeminist ideas and desire for peaceful and harmonious interactions between men and women, as well as people and the public environment. As a result, an ecofeminist reading of the text clarifies the book's complicated public environment and gender concerns.

### 4.2. The Ideal Relationship from the Perspective of Ecofeminism

There were many vivid depictions of public environments in Lawrence's childhood, which may be observed in his novel. Public environment was destroyed as a result of the Industrial Revolution. Lawrence began to condemn men's actions and called for preserving public environment after witnessing his beloved environment being destroyed. Lawrence was influenced by several women during his life. He admired them. However, women had no status during his age. Many women participated in women's movements to fight for their rights. Lawrence supported the women's movements after being influenced by his female acquaintances. In Sons and Lovers, Lawrence combined themes of environmental protection with issues of women's rights protection. Lawrence's concepts were in line with ecofeminism's principles, despite the fact that ecofeminism had not yet been proposed. His ecofeminist notion was portrayed by his views in the novel.

Lawrence attempted to awaken human beings' awareness of ecofeminism by depicting the oppression of women and environment, demonstrating the specific relationship between both. Lawrence described the ideal relationship between women and public environment as one of harmony, peace, and love, and he encouraged humans to create this kind of ideal relationship.

Men in Sons and Lovers desired to master public environment, but men's inner selves yearn for it as well. Patriarchy refers to the male-dominated framework of modern culture and political institutions. Women's rights are thought to be jeopardized by such arrangements. However, it has been noted that patriarchal systems of government do not benefit all men of all classes. The exploiters' desire for property outweighed their desire for a healthy environment. The working class had no choice but to take whatever came their way and labored to make a living.

Men and women should have common topics, and should communicate with each other. The status between them should be equal, not be oppressed. In addition, they should have harmonious sexual life and spiritual communication. Lawrence held the opinion that there was no need to yoke them with any bond at all. The only morality is to have man true to his manhood, woman to her womanhood, and let the relationship form by itself, in all honor. Therefore, the ideal relationship between man and woman should be that “both are equal, two in one complete.” A couple should be equal and love each other, they should depend on each other, overcome the differences of culture background and the difficulties in life together, raise children together, and spend life together.

Throughout his life, Lawrence was concerned about the links between women and public environment, men and public environment, and women and men. He loved the environment. Public environment was well described in Sons and Lovers. However, the Industrial Revolution had an impact on his hometown. He saw the damaged landscapes and the vanishing woods. He was also witness to men-women confrontations. As a result, he pushed for the preservation of environment and the liberation of women. He maintained that public environment, men, and women should all live in harmony. This subsection will discuss the ideal relationships from the perspective of ecofeminism, as well as the origins of Lawrence's ideas.

Lawrence's enthusiasm for the environment was primarily influenced by his father, Arthur Lawrence, who was passionate about wildlife and knew a lot about it. He would occasionally bring flowers or animals home and tell his children their names. He would tell his children about the plants and animals when they went on a walk outside. Lawrence had a natural passion for the public environment since he was a youngster, due to his father's influence. The Chambers relocated to the Haggs Farm as teenagers, and Lawrence paid them regular visits. He was enamored by gardens, houses, trees, flowers, and the countryside.

Lawrence embraced certain feminist ideals as a result of female influence. These women's images served as models for the heroines in his novels. He was a strong supporter of women's rights movements. He did not like dominant women who wanted to be in charge of everything. He advocated for women to have the same rights, position, and opportunities as males. On the other hand, he did not support women discriminating against men. In his opinion, men and women should depend on each other. Moreover, Lawrence hopes for a harmonious relationship filled with love among the three—men, women, and public environment.

Lawrence's views on the interactions between men and environment, as well as men and women, are ecofeminist. Ecofeminists believe that women and public environments have a direct relationship. The patriarchal culture, which holds women and public environment to be inferior to males, is the basis of the same oppressive condition. This system defends men's dominance and women's subjection to public environment. Thus men are the masters of all things, while women and public environment should obey the orders from men. The same oppression makes women and public environment unite together.

Ultimately, Sons and Lovers is a masterpiece in which Lawrence expresses his concern for men's, women's, and natural connections. Lawrence hopes to raise public awareness about the need of protecting environment and women. The current climate is peculiar, and the entire world is constantly threatened by global economic and ecological crises. Therefore, rereading Sons and Lovers from an ecofeminist viewpoint is extremely important. This novel inspires us to create a future in which men, women, and public environment all enjoy healthy and peaceful interactions. Thus, we can establish a nice public environment in this way.

## 5. Conclusion

Taking the isomorphism between nature and women as a logical starting point, ecofeminists have profoundly expounded that the root of ecological crisis is closely related to patriarchal culture. The emergence and meaning of ecofeminism are rights and promises, and its ultimate goal and ideal is to strive for the equality and harmonious development of men and women. Ecofeminism has a unique rational thinking and new insights, and its logical methodology is from heroic ethics to comprehensive ethics. As the pioneer of public environmental protection, women have made great contributions to the common liberation of public environment and women. As the practice pioneer of public environmental protection, women have made great contributions to the public environment and the common liberation of women. Public environmental protection affected by ecological feminism was initially a conscious individual mobilization behavior caused by worrying about family life. After entering the middle of the 20th century, under the sustained reporting, shaping, and mobilization of the foreign mass media, public environment protection began to gradually move to the public stage, connect with the issue of justice, promote a wave of social movement involving the whole people, and ultimately exceed the limits of the national framework. In the process of women's public environmental protection, their understanding of nature has undergone a transformation from “housekeeping” nature to ecological nature, reflecting their strong potential and power in public environmental protection. Women's involvement and participation in public environmental issues is their attempts and efforts to enter the public domain, resist patriarchy, and change social status. They show society a unique perspective to solve public environmental issues by respecting differences and diversity, which provides a new path for women to participate in public affairs and realize their own liberation, and also provides a way for countries around the world to deal with national and social issues.

## Figures and Tables

**Figure 1:** Schematic diagram of ecofeminism.

**Figure 2:** Whole context for ecofeminism.

## Data Availability

All data used to support the findings of the study are included within this paper.

## References

[1] Arjona E. M. (2019). Ecofeminism and interculturality. *FEMINISMO-S*.

[2] Mallory C. (2013). Environmental justice, ecofeminism, and power, linking ecology and ethics for a changing world: values, philosophy. *Action*.

[3] Gonzalez G. A. T. (2017). The critical ecofeminism of alicia puleo: weaving the thread of the “new ariadna”. *Investigaciones Feministas*.

[4] Gao X. X. Critical analysis of “nature-women” metaphor from ecofeminism.

[5] Gough A., Whitehouse H. (2020). Challenging amnesias: re-collecting feminist new materialism/ecofeminism/climate/education. *Environmental Education Research*.

[6] Ekinci E. Ecofeminism in the context of women and ecology.

[7] Ding Z. R. Comparative study of ecofeminism in Chinese and western feminist literature.

[8] Zhao Y. S., Xiong Y., Li L. J. (2018). Appreciation of william and dorothy wordsworth from ecofeminism perspective, 3RD international conference on education and social development. *ICESD 2017)*.

[9] Qiu Y. (2021). From androcentrism to ecofeminism: gary snyder’s goddess worship. *ORBIS Litterarum*.

[10] Laplonge D. (2016). Exploring the distance between ecofeminism and women in mining (WIM). *Extractive Industries and Society*.

[11] Wang W. H. (2008). Rereading jane eyre from the perspective of ecofeminism. *Foreign Literature Studies*.

[12] Devika J., Caregiver V. S. (2010). Citizen? reflections on ecofeminism from Kerala state, India. *Man in India*.

[13] Mallory C. (2013). Locating ecofeminism in encounters with food and place. *Journal of Agricultural and Environmental Ethics*.

[14] Wei Q. Q. (2018). Toward a holistic ecofeminism: a Chinese perspective. *Comparative Literature Studies*.

[15] A G Oliveira F. (2019). The sexist diet: contributions from critical ecofeminism for a decolonialization of the palate. *Question*.

[16] Njoh A. J., Ayuk-Etang E. N. M. (2021). Determinants of ecofeminism in anglophone cameroon: a pestech analysis. *Journal of Asian and African Studies*.

[17] Wang X. Y. Women and construction of an ecological civilization from the perspective of ecofeminism.

[18] Rocha R. K. d., Feldman A. K. T., Silva M. C. (2020). Ecocrítica e ecofeminismo: uma leitura do conto “A porca”. *Revista Ártemis*.

[19] Konik I. (2018). Ubuntu and ecofeminism: value-building with african and womanist voices. *Environmental Values*.

[20] Gu X. Challenges and public participation strategies on coastal resources protection in China.

[21] Bartniczak B. (2011). State Aid in Environment Protection in Scandinavian Countries. *Hradec Economic Days*.

[22] Liu Y. X. On universal design methods focusing on environment resources protection.

[23] Kauder B., Potrafke N., Ursprung H. (2018). Behavioral determinants of proclaimed support for environment protection policies. *European Journal of Political Economy*.

[24] Yang Z. F., Li Q. L. Research on the construction of social co-governance system of ecological environment protection.

[25] Han Q. F., Ge S. L., Yu J. L. The relationship between ecological environment protection and social development to Chinese resource-exhausted cities.

[26] Kings S. E. (2017). Intersectionality and the changing face of ecofeminism. *Ethics and the Environment*.

[27] Wei Q. Q. (2014). “Staying female while knowing male”: a new interpretation of ecofeminism in a cross-cultural context. *Foreign Literature Studies*.

[28] Klemmer C. L., McNamara K. A. (2020). Deep ecology and ecofeminism: social work to address global environmental crisis. *Affilia*.

[29] Gaard G. (2015). Ecofeminism and climate change. *Women’s Studies International Forum*.

[30] Bravo M. A. B. (2016). Ecofeminism: a new way to look at nature. *Arbor-Ciencia Pensamiento y Cultura*.

[31] Li D. (2013). Ecofeminist literary criticism in mainland China: a window into China’s academic globalization. *Asian Women*.

[32] Liu Y., Anser M. K., Zaman K. (2021). Ecofeminism and natural resource management: justice delayed, justice denied. *Sustainability*.

[33] Wang M. Y. An analysis of ideology in D. H. Lawrenc’s sons and lovers.

